The article "Characterising Vascular Cell Monolayers Using Electrochemical Impedance Spectroscopy and a Novel Electroanalytical Plot" was retracted in 2021. Reasons: no approval from the institution; no approval from a third party; a breach of policy by an author.

# Characterising Vascular Cell Monolayers Using Electrochemical Impedance Spectroscopy and a Novel Electroanalytical Plot

**DOI:** 10.2147/NSA.S266663

**Published:** 2020-09-23

**Authors:** Anubhav Bussooa

**Affiliations:** 1 BHF Cardiovascular Research Centre, University of Glasgow, Glasgow G12 8TA, UK

**Keywords:** impedance sensors, electrochemical impedance spectroscopy, Bode plot, Nyquist diagram, electroanalytical plot

## Abstract

**Introduction:**

Biological research relies on the culture of mammalian cells, which are prone to changes in phenotype during experiments involving several passages of cells. In regenerative medicine, specifically, there is an increasing need to expand the characterisation landscape for stem cells by identifying novel stable markers. This paper reports on a novel electric cell-substrate impedance sensing-based electroanalytical diagram which can be used for the “electrical characterisation” of cell monolayers consisting of smooth muscle cells, endothelial cells or co-culture.

**Materials and Methods:**

Interdigitated electrodes were microfabricated using standard cleanroom procedures and integrated into cell chambers. Electrochemical impedance spectroscopy data were acquired for 2 vascular cell types after they formed monolayers on the electrodes.

**Results and Discussion:**

A Mean impedance per unit area vs Mean phase plots provided a reproducible, visually obvious and statistically significant method of characterising cell monolayers. This electroanalytic diagram has never been used in previous papers, but it confirms findings by other research groups using similar approaches that the complex impedance spectra of different cell type are different. Further work is required to determine whether this method could be extended to other cell types, and if this is the case, a library of “signature spectra” could be generated for “electrical characterisation” of cells.

## Introduction

Biological research relies on the culture of mammalian cells, which are prone to changes in phenotype during experiments involving several passages of cells.^1^ The non-homeostatic culture conditions in culture flasks, which is subject to sudden changes of culture medium, inhibit cells from terminally differentiating and promotes maintenance of phenotypic flexibility.^2^,^3^ During standard cell culturing, there is lack of demand for specific cell functionalities leading to loss of their expression. Moreover, there is an alarming rate of cross-contamination of human cell lines with other cells, such as HeLa cells, and with microorganisms, such as mycoplasma.^4^,^5^ When such discrepancies go unnoticed, erroneous results are generated and this contributes to the multi-billion dollar irreproducibility problem.^1^ On the other hand, controlled modification of biochemical and biomechanical microenvironment can induce stem cell differentiation towards specific phenotypes.^6^ A range of biochemical assays are used to characterise stem cells at the molecular level.^7^ However, these assays involve fixing, staining, detaching, lysing or fluorescent-labelling of the stem cells, which thus precludes their therapeutic potential. Overall, there is a need for in situ, label-free and non-invasive characterisation of the phenotypes of human cell lines and stem cells.

The article "Characterising Vascular Cell Monolayers Using Electrochemical Impedance Spectroscopy and a Novel Electroanalytical Plot" was retracted in 2021. Reasons: no approval from the institution; no approval from a third party; a breach of policy by an author.

Electric Cell-substrate Impedance Sensing (ECIS) is a well-established, label-free and non-invasive electroanalytical tool, which is used to monitor adherence, proliferation, migration and death of adherent cells, but its full potential for “electrical characterisation” of different cell types had not been fully explored.^8^ ECIS was pioneered by Nobel Laureate Ivar Giaever and Charles Keese.^9^ The ECIS electrodes are co-planar, that is, integrated onto the same 2D surface, usually the bottom of cell culture chambers. Adherent cells are grown directly on the electrodes.^10^ The system is operated by applying a AC signal of 1 µA through a constant current source at various frequencies.^9^ The in-phase and out-of-phase voltage data are recorded and from these the impedance data is outputted. Adherence of cells to the electrodes disrupts the electrode/electrolyte interface, causing large increases in impedance. The ECIS electrodes are scalable and the sensitivity of detection increases with decrease in electrode surface area.^11^ Zhang et al found that miniaturising the electrodes significantly increased the detected change in impedance.

Most attempts for classifying cell lines through ECIS data were carried out using the impedance measurement at a single frequency over a large time period.^8^ Using this method, different research groups found that different cell lines could be distinguished by the fact that impedance v/s time curve peaked higher or increased more rapidly.^12^,^13^ Most ECIS experiments are carried out at single frequency (traditionally 4 kHz), implying that valuable information obtained at other frequencies are overlooked.^8^ Gelsinger, Tupper and Matteson (2019) carried out a meta-analysis of ECIS studies and used advanced mathematical techniques to develop a classification method for 15 different cell lines. They found that plotting the maximum resistance (32 kHz) against resistance at 2 h (32 kHz) and the maximum resistance (16 kHz) against resistance at 2 h (64 kHz) were the most promising methods for ECIS-based cell classification.

The article "Characterising Vascular Cell Monolayers Using Electrochemical Impedance Spectroscopy and a Novel Electroanalytical Plot" was retracted in 2021. Reasons: no approval from the institution; no approval from a third party; a breach of policy by an author.

Electrochemical Impedance Spectroscopy (EIS) is another impedance-based method, which is less commonly used in medical research, compared to ECIS. It is another powerful technique used to analyse the complex electrical impedance of a system, which is sensitive to changes in bulk properties and surface phenomena (Lisdat and Schäfer, 2008). It is used for antibody, enzyme, DNA and cell sensing. In contrast to ECIS, this technique involved measurement of impedance over a large frequency range (sweep). EIS enables the optimal frequency, at which the relative changes are highest, to be determined. The impedance spectra generated allows the characterisation of layers, surfaces or membranes. The results of EIS are represented using Bode plots and Nyquist plots (Moisel, de Mele and Müller, 2008). For the Bode plot, the magnitude of the impedance (│Z│) and the phase angle (θ) are plotted against the logarithm of the frequency. The real impedance (Z’) and imaginary impedance (Z”) are related to its magnitude (│Z│) and phase (θ) by the following equations:

1 $${\rm{Real \ impedance }}\left({Z'} \right){\rm{ = }}\left| Z\right|\,{\rm{ Cos \theta }}$$

2 $${\rm{Imaginary \ impedance }}\left({Z''} \right){\rm{ = }}\left| Z\right|\,{\rm{Sin \theta }}$$

For the Nyquist plot, the negative of the imaginary impedance is plotted against the real impedance.^14^ Each data point represents the complex impedance at one frequency. Semi-circles in the Nyquist plot indicate a barrier of the charge transfer process or an insulating electrode surface. When EIS is used to characterise biological tissue (Figure 1), 2 main components are generally identified: the electrode/tissue interface (which dominates at low frequencies) and the tissue impedance (which dominates at high frequencies).^15^ The Nyquist plot allows these 2 phenomena to be clearly visualised.

**Figure 1:** Typical Nyquist plot of electrode/tissue interface, showing 2 depressed semi-circular arcs. © [2015] IEEE. Reprinted, with permission, from Lewis N, Lahuec C, Renaud S, et al. Relevance of impedancespectroscopy for the monitoring of implant-induced fibrosis:a preliminary study. In: IEEE Biomedical Circuits and Systems Conference: Engineering for Healthy Minds and Able Bodies,BioCAS 2015 – Proceedings; 2015; Institute of Electrical andElectronics Engineers Inc.15)

Non-destructive verification of the appropriate phenotypes is important in stem cell differentiation studies.^7^ Bagnaninchi and Drummond used EIS to monitor adipose-derived stem cell differentiation. They used complex plane analyses to characterise the cells at early and late differentiation. They found that the Log Resistance v/s Log Reactance curves were significantly different between osteo-induced and adipo-induced stem cells. They hypothesised that this difference was due to the appearance of specialised functions: formation of lipid droplets for adipocytes and production of mineralized matrix for osteo-induced cells. Zhang et al^16^ also used EIS to distinguish between skin cancer cells and normal cells. The resistance and capacitance of the cell layer covering the working electrode was plotted against the cell number. They found that the resistance of the cancer cells was significantly lower than that of the normal cells, while the capacitance was not significantly different. Teixeira et al^17^ carried out EIS using a 4-terminal setup to distinguish mouse fibroblasts (L929) from human keratinocytes (HaCaT). On a Nyquist diagram, L929 showed only one dispersion while HaCaT showed 2 dispersions, indicated by 2 semi-circles. In another paper,^18^ the same research group found that on a Nyquist diagram, the curves for cancerous tissues formed a separate cluster from curves for normal tissue. Guo et al^19^ used EIS methods for in vitro monitoring of a human hepatocarcinoma cell line, grown on indium tin oxide semiconductor slides. They used a frequency range of 0.01 Hz to 100 kHz and analysed their results using Nyquist plots. At very low frequencies, the real component and imaginary components of the impedance had a linear relation, representing the diffusion-limited electron-transfer process. At low frequencies, the relation was semi-circular, representing the electron-transfer-limited process. At high frequencies, part of the high-frequency semi-circular arc could also be observed.

The article "Characterising Vascular Cell Monolayers Using Electrochemical Impedance Spectroscopy and a Novel Electroanalytical Plot" was retracted in 2021. Reasons: no approval from the institution; no approval from a third party; a breach of policy by an author.

In regenerative medicine, there is an increasing need to expand the characterisation landscape for stem cells by identifying novel stable markers.^20^,^21^ The inconsistencies in isolation and expansion methods of stem cells lead to variations in cell phenotypes. It is crucial that the appropriate cells, expressing the appropriate phenotypes, are used to engineer biological tissue and the phenotypes and cell localisations are maintained until the engineered tissue is implanted or used for drug screening. For example, when engineering living tubular vascular grafts, it is critical that the inner layer consists of a confluent endothelium, as this offers a non-thrombogenic interface with blood, and that the outer later consists of smooth muscle tissues, which can relax and contract to withstand haemodynamic stress.^22^–^27^

To the author’s knowledge, there are no previous studies which have used EIS for the “electrical characterisation” of smooth muscle cells and endothelial cells. In this paper, a novel electroanalytic diagram (mean impedance per unit area v/s mean phase) was used to distinguish smooth muscle cells, endothelial cells and a co-culture of these 2 cell types. Area under the curve analysis showed a statistically significant difference between the different cell populations. The paper also demonstrates the inefficiency of the commonly used Bode diagrams for characterising and distinguishing different vascular cell types. This novel method of electrical characterisation of vascular cells could be valuable in engineered vascular grafts. It could be used to non-invasively determine whether endothelial cell only and smooth muscle cells only are located in the inner and outer layers, respectively, of the engineered grafts. Even though only vascular cell types were used in this paper, it is possible that this method could be used to distinguish between other cell types (e.g. cancer cells and non-cancer cells) and to monitor differentiation of stem cells towards different phenotypes.

The article "Characterising Vascular Cell Monolayers Using Electrochemical Impedance Spectroscopy and a Novel Electroanalytical Plot" was retracted in 2021. Reasons: no approval from the institution; no approval from a third party; a breach of policy by an author.

## Materials and Methods

### Microfabrication and Experimental Setup

Interdigitated electrodes (IDEs) were microfabricated within the James Watt Nanofabrication Centre of University of Glasgow, using standard microfabrication techniques. A custom-designed photolithographic mask containing 2 different sizes of IDE was used. The Large IDE (LIDE) had an electrode surface area of 28.8 mm^2^ and consisted of 2 sets of 20 fingers, each with the following dimensions: length 800 µm, width 100 µm and 100 µm separation between each finger. The LIDE was miniaturised by a linear factor of 4 (area factor of 16) in order to generate the SIDE. The SIDE had an electrode surface area of 1.8 mm^2^ and consisted of 2 sets of 20 fingers, each with the following dimensions: length 200 µm, width 25 µm and 25 µm separation between each finger. The electrodes were screen printed on microscope slides (Sigma Aldrich, UK) and consisted of 100 nm thick gold layer with 10 nm titanium adhesion layer. Using UV curable glue (Loctite, Germany), plastic chambers from a commercially available slide chamber (Sigma Aldrich, UK) were mounted onto the screen printed glass slide (Figure 2). Electrical wires were soldered to the contact pads of the LIDE and SIDE. The experimental setup (Figure 3) consisted of an LCR meter (Hioki IM 3536, Japan) which was interfaced using a PC. The IDEs were connected to the LCR meter for impedance measurements.

**Figure 2:** Photograph of cell culture chamber containing large IDE and small IDE.

**Figure 3:** Experimental setup consisting of microfabricated cell chambers connected to the LCR meter, which is interfaced using a PC.

### Primary Cell Culturing and Cell Seeding

Mouse Aortic Smooth Muscle Cells (MASMC) and immortalised murine endothelial cells (sEND1) were used in the experiments for this research paper. No direct experiments with animals were carried out. MASMC had previously been isolated and characterised by Mercer et al,^28^ where all animal experimental procedures conformed to animal Ethical Committee approval and UK Home Office licensing. sEND1 had previously been transfected and characterised by Leiper et al.^29^ The cells were cultured in DMEM media (Sigma Aldrich, UK) supplemented with 10% Foetal Bovine Serum in culture flasks. Once sub-confluent, the cells were trypsinised and 400,000 cells were then seeded into the fabricated device, and the cell suspension was pipetted up and down a few times to ensure a homogeneous population was plated. Pure MASMC populations, pure sEND1 populations and co-culture (1:1 ratio) were used in separate experiments. The LIDE and SIDE were present within the same cell chamber. Thus, the same cell monolayer covered the LIDE and the SIDE.

The article "Characterising Vascular Cell Monolayers Using Electrochemical Impedance Spectroscopy and a Novel Electroanalytical Plot" was retracted in 2021. Reasons: no approval from the institution; no approval from a third party; a breach of policy by an author.

### Electrochemical Impedance Spectroscopy

The microfabricated cell chambers were sterilised by misting with 70% ethanol and rinsing with deionised water. The LCR meter (IM3536 – Hioki, Japan) was used in the constant current (CC) mode, with the current set at 10 µA. The baseline impedance spectra for the frequency range 10 Hz to 1 MHz were first measured with DMEM culture medium only. Then, 400,000 cells were seeded into the chambers and allowed to adhere to the bottom (glass + electrodes) of the chambers for 18 h, inside an incubator (37°C and 5% CO_2_). Microscopic observation in prior experiments showed that this cell number ensured that the cells formed a confluent monolayer at 18 h. Then, the experimental impedance spectra, with the cells, were acquired. Complex impedance is a vector quantity and in this paper, impedance refers to the magnitude of the impedance and phase refers to its direction. In order to compare between the Large IDE and Small IDE, the impedance was normalised to impedance per unit area. As complex impedance is a vector quantity, only the magnitude of the impedance is dependent on the area of the electrode while the phase is independent of the area of the electrode. Hence, normalisation was carried out by dividing the magnitude of the impedance by the area of the respective electrodes and keeping the phase constant.

### Data Collection & Statistical Analysis

The impedance spectra were recorded using the LCR meter with 3 technical replicates (3 microfabricated chambers) for the 3 cell populations (MASMCs, sEND1 and co-culture). All data in the graphs are representative of replicate data samples with a mean ± standard deviation (SD). Area Under Curve (AUC) was used to analyse the Mean impedance per unit area (MIPUA) vs Frequency plots (Figure 4) and the Mean impedance per unit area (MIPUA) vs Mean phase plots (Figure 5). The comparison was carried out in 2 ways:

1. Between the same cell populations (MASMC, sEND1 and co-culture) and different electrodes (LIDE & SIDE).
2. Between the same electrode types and different cell populations.

The article "Characterising Vascular Cell Monolayers Using Electrochemical Impedance Spectroscopy and a Novel Electroanalytical Plot" was retracted in 2021. Reasons: no approval from the institution; no approval from a third party; a breach of policy by an author.

For the MIPUA vs Frequency plots, the AUC increase was calculated by subtracting the AUC of the “culture medium only” curve from the AUC of the “culture medium + cells” curve. The AUC increase was compared between different pairs of cell populations and electrode types using One-way ANOVA. For the MIPUA vs Mean phase plots, AUC were measured for “culture medium + cells” curves for the range 1–10 Ω/mm^2^ for LIDE and for the range 100–1000 Ω/mm^2^ for SIDE. AUC was compared between different pairs of cell populations for the different electrode types using Student’s *t*-test. Statistical significance was displayed as p < 0.05 (*), P < 0.01 (**) or P < 0.001 (***). All analyses were performed and plotted using GraphPad Prism (v 5).

**Figure 4:** Mean impedance per unit area vs Frequency and Mean phase vs Frequency spectra acquired using Large IDE with MASMC (**A**), sEND1 (**B**) & co-culture (**C**) and using Small IDE with MASMC (**D**), sEND1 (**E**) & co-culture (**F**).

**Figure 5:** Mean impedance per unit area vs Mean phase plots acquired using Large IDE with MASMC (**A**), sEND1 (**B**) & co-culture (**C**) and using Small IDE with MASMC (**D**), sEND1 (**E**) & co-culture (**F**).

## Results and Discussion

**Figure 6:** MASMCs and sEND1 in suspension within the electrode area immediately after seeding at 0 h and formation of cell monolayers at 18 h.

In Figure 6, bright-field images of MASMC and sEND1 at 0 h (just after seeding into the chambers) are shown. At this timepoint, the cells are rounded and in suspension around the electrode area. Images of the cells at 18 h are also shown. At this timepoint, the cells have spread on the electrodes and formed a monolayer.

### Bode Plots

The MIPUA vs Frequency and Mean Phase vs Frequency spectra (Bode Plots) for MASMC, sEND1 and co-culture (1:1 ratio) cell populations recorded using LIDE and SIDE are shown as individual graphs in Figure 4. The Bode plots for MASMC, sEND1 and co-culture are also shown on the same graph for LIDE (Supplementary Figure 5) and for SIDE (Supplementary Figure 6). The impedance spectra and the phase spectra with culture medium only (baseline) are shown as red dots and purple triangles, respectively. The impedance spectra and the phase spectra with culture medium + cells (experimental) are shown as blue dots and blue-green triangles, respectively. For the LIDE, the experimental phase spectra is above the baseline between approximately 1 kHz and 10 kHz and below the baseline >10 kHz. For the SIDE, the experimental phase spectra is above the baseline between approximately 100 Hz and 100 kHz and below the baseline >100 kHz. The impedance spectra diverge between approximately 1 kHz and 1 MHz for the LIDE, which indicates its optimum sensing frequency range. The impedance spectra diverge between approximately 1 kHz and >1 MHz for the SIDE, which indicates its optimum sensing frequency range. The frequency sweep range of the LCR had a maximum of 1 MHz, and thus the upper end of the optimum frequency range for the SIDE could not be determined. However, this shows that miniaturising the IDE shifts the frequency parameters for cell sensing.

The article "Characterising Vascular Cell Monolayers Using Electrochemical Impedance Spectroscopy and a Novel Electroanalytical Plot" was retracted in 2021. Reasons: no approval from the institution; no approval from a third party; a breach of policy by an author.

A second method of normalisation was also used. The experimental data with cells was normalised to the baseline data without cells by dividing the individual experimental impedances by the individual baseline impedance at the corresponding frequency. The “Baseline Normalised” Impedance vs Frequency curves for MASMC, sEND1 and co-culture with LIDE and SIDE are shown in Supplementary Figure 2. AUC and Student’s *t*-test analysis was carried out, and these results are shown in Supplementary Figure 3.

**Figure 7:** AUC increase of the Impedance v/s Frequency curves for the MASMC, sEND1 and co-culture with LIDE and SIDE(p < 0.05 (*), p < 0.01 (**) & p < 0.001 (***)).

Within the optimum frequency range, the experimental impedance spectra is higher than the baseline impedance spectra, for both LIDE and SIDE, indicating an increase in impedance due to cell adhering to the electrodes. AUC analyses (Figure 7) showed that impedance increase detected by the SIDE, compared to LIDE, is significantly higher for all of MASMC, sEND1 and co-culture. This implied that, for the same cell monolayer, the SIDE can detect a higher increase in impedance per unit area compared to LIDE. Thus, miniaturising the IDE increases its detection capability. At equal cell densities, the impedance increase detected by SIDE was significantly higher for MASMC compared to sEND1 and for co-culture compared to sEND1. The impedance increase detected by LIDE was not significantly different for any of the cell populations. This implies that SIDE can detect differences in the impedance magnitude increase generated by equal cell densities. Thus, EIS measured using the SIDE could be potential method of characterising vascular cell monolayers. Overall, normalising the impedance to the unit area (Figures 4 and 7) allowed more cell populations to be distinguished, compared to normalising the experimental impedance to the baseline (Supplementary Figures 2 and 3).

The article "Characterising Vascular Cell Monolayers Using Electrochemical Impedance Spectroscopy and a Novel Electroanalytical Plot" was retracted in 2021. Reasons: no approval from the institution; no approval from a third party; a breach of policy by an author.

This difference could be due to differences in the innate electrical properties of the cells or in cell/electrode interface of the MASMC and sEND1. Mamouni and Yang (2011)^30^ used Interdigitated Electrodes to distinguish between a non-cancer oral epithelial cell type and an oral cancer cell type. They found that, at equal cell numbers, the non-cancer cells generated a smaller magnitude of impedance compared to the cancer cells. My findings are in line with theirs, as at equal cell densities, sEND1 generated a lower increase in impedance compared to MASMC. The increase in impedance is, however, also proportional on the cell density.^31^ A low cell density of MASMC could thus produce a similar impedance spectrum as a high cell density of sEND1. Hence, distinguishing cell types based on impedance spectra would only be possible at identical cell densities. Ensuring equal cell densities is usually difficult because of the natural biological variations of cells. Different cell types generate impedance spectra with identical shapes, and thus Bode plots are not suitable for characterising different cell types. Other electroanalytical diagrams should be used for this purpose.

### Characterising Electrode/Tissue Interface Using Nyquist Plots

The LCR meter used outputs the following data: frequency, magnitude of impedance (│Z│) and phase (θ). In order to plot Nyquist diagrams, the real and imaginary impedances were calculated using Equations 1 and 2. The real and imaginary impedances were normalised by dividing by the surface area of the respective electrodes, 28.8 mm^2^ for LIDE and 1.8 mm^2^ for SIDE. The Nyquist plots for SIDE seeded with MASMC and sEND1 are shown in Figure 8. The Nyquist plots for all the cell populations and electrode types are shown in Supplementary Figure 1. The red dots represent the complex impedance of the electrodes + medium (baseline) while the blue dots represent the complex impedance of electrodes + medium + cells (experimental). The complex impedance followed a depressed semi-circular arc, as shown in Figure 1. Adherence of cells on the electrodes caused a deviation of the experimental curve from the baseline curve. The impedance measurements were carried out for the frequency range of 10 Hz to 1 MHz, because this was the full range of the LCR meter used.

Guo et al^19^ observed a linear relation between real and imaginary components of impedance at very low frequencies, a first semi-circular relation at low frequencies and a second semi-circular relation at high frequencies. They used a frequency range of 0.01 Hz to 100 kHz. In my experiments, the linear relation was not observed because the lowest frequency was 10 Hz. Even though I carried out measurements up to 1 MHz, the semi-circular relation was not observed. This could be due to differences in the baseline impedance of the electrodes used. In my experiments, gold interdigitated electrodes were used, while in their experiments indium tin oxide electrodes were used. The Nyquist plots for SIDE with MASMC (Figure 8A) and sEND1 (Figure 8B) have similar shapes, and thus do not allow a visually obvious distinction between these 2 cell types. This was also the case with LIDE (Supplementary Figure 1).

The article "Characterising Vascular Cell Monolayers Using Electrochemical Impedance Spectroscopy and a Novel Electroanalytical Plot" was retracted in 2021. Reasons: no approval from the institution; no approval from a third party; a breach of policy by an author.

**Figure 8:** Nyquist plots for Small IDE with MASMC (A) and sEND1 (B).

### Distinguishing Cell Types Using Mean Impedance per Unit Area vs Mean Phase Plot

In this section, the Mean impedance per unit area (MIPUA) was plotted against the mean phase (Figure 5) for MASMC, sEND1 and co-culture with Large IDE and Small IDE. The curves for MASMC, sEND1 and co-culture were shown on the same graph for LIDE (Supplementary Figure 7) and SIDE (Supplementary Figure 8). For each graph, most of the data points were in the 4th quadrant, whereas with the Nyquist plots (Figure 8), most data points are in the 1st quadrant. This is simply because the Nyquist diagrams are plotted with real component of impedance on the x-axis and negative of the imaginary component of impedance on the y-axis. In Figure 5, the red curves represent the electrodes + medium (baseline). In all 6 plots (Figure 5A–F), they can be described as decay curves. The blue curves represent the electrodes + medium + cells (experimental). For both LIDE (Figure 5B) and SIDE (Figure 5E), the blue curves with sEND1 can also be described as decay curves. The blue curves with MASMC and co-culture for both LIDE (Figure 5A and D) and SIDE (Figure 5C and F) are different from the sEND1 decay curves. A “bulge” is observed in the blue curves between a MIPUA of 1–10 Ω/mm^2^ for LIDE and 100–1000 Ω/mm^2^ for SIDE, as indicated by the black dashed lines. Thus, a pure sEND1 population of 400,000 generated decay curves with both LIDE and SIDE, while a pure MASMC population of 400,000 generated “bulged” curves with both LIDE and SIDE.

**Figure 9:** AUC for Mean impedance per unit area vs phase diagrams for culture medium+cells curves for the real impedance per unit area range 1–10 Ω/mm^2^ for LIDE and 100–1000 Ω/mm^2^ for SIDE( p < 0.05 (*), p < 0.01 (**) & p < 0.001 (***)).

Interestingly, a co-culture of 200,000 sEND1 + 200,000 MASMC also generated “bulged” curves with both LIDE and SIDE. The “bulge” is most likely due to the MASMC in the co-culture, implying that the electrodes can detect MASMC even within a co-culture. Further experiments are required to determine the lowest MASMC to sEND1 ratio which would still generate this characteristic “bulge”. Thus, this “bulge” in the experiment curve provides a visually obvious method of distinguishing the different cell populations. Area Under the Curve (Figure 9) was used to analyse the MIPUA vs Mean phase plots. As the “bulge” was located between a MIPUA of 1–10 Ω/mm^2^ for LIDE and 100–1000 Ω/mm^2^ for SIDE, AUC analysis was only carried out for these ranges for the experimental (blue) curves. The AUC was compared between different pairs of cell populations for LIDE and SIDE using Student’s *t*-test. For the LIDE, the AUC was significantly different for MASMC and sEND1. For SIDE, the AUC was significantly different from all of the cell population combinations. This demonstrates that the SIDE is more sensitive than LIDE for characterising different vascular cell monolayers.

The article "Characterising Vascular Cell Monolayers Using Electrochemical Impedance Spectroscopy and a Novel Electroanalytical Plot" was retracted in 2021. Reasons: no approval from the institution; no approval from a third party; a breach of policy by an author.

### Mean Impedance per Unit Area vs Mean Phase Plot Curve Fitting

Origin 2020b Version 9.7.5.184 (OriginLab Corporation – USA) was used for curve fitting of the individual blue experimental curves (representing electrodes + medium + cells) from Figure 8, using the following “Three-phase exponential decay function with time constant parameters”:

$$y = {y_0} + {A_1}{e^{ - {x \over {{t_1}}}}} + {A_2}{e^{ - {x \over {{t_2}}}}} + {A_3}{e^{ - {x \over {{t_3}}}}}$$

One example of the curve fitting for each combination (cell types and electrode types) is shown in Figure 10. The blue data points represent the experimental data and the green line represents the data fitted using the above equation. The curve parameters y_0_, A_1_, t_1_, A_2_, t_2_, A_3_ & t_3_ and the r^2^ value were determined for all the 3 replicates of each combination. The mean and standard deviation was calculated and pair-wise Student’s *t*-test. These results are shown in Table 1 (LIDE) and Table 2 (SIDE).

**Table 1:** Curve Fitting Parameters and R^2^ Value for MIPUA Vs Mean Phase Curve Acquired Using LIDE

Large IDE							
	MASMC		sEND1		Co-Culture		Student’s *t*-Test
	Mean	SD	Mean	SD	Mean	SD	
r^2^	0.99947	0.00023	0.99825	0.00230	0.99891	0.00125	ns
y0	−83.98954	4.03106	−3.75239E+06	6.49918E+06	−79.88563	6.47046	ns
A1	2.87973E+04	4.70371E+04	115.51728	102.41076	2.55126E+09	4.41886E+09	ns
t1	0.12891	0.04190	2.03947	2.90784	0.09525	0.07091	ns
A2	60.84396	8.17751	76.13780	29.76812	155.29689	166.86816	ns
t2	4.70275	0.55474	1.63647	0.88305	2.63877	2.08102	** (for MASMC v/s sEND1)
A3	16.27912	2.19167	3.75232E+06	6.49916E+06	33.29552	22.77927	ns
t3	25.18145	7.95958	1.02326E+08	1.77234E+08	15.33905	9.95537	ns

**Notes:** Statistical significance is indicated as ns (not significant). *p-value < 0.05, **p-value < 0.01 and ***p-value < 0.001.

The article "Characterising Vascular Cell Monolayers Using Electrochemical Impedance Spectroscopy and a Novel Electroanalytical Plot" was retracted in 2021. Reasons: no approval from the institution; no approval from a third party; a breach of policy by an author.

**Table 2:** Curve Fitting Parameters and R^2^ Value for MIPUA vs Mean Phase Curve Acquired Using SIDE

Small IDE							
	MASMC		sEND1		Co-Culture		Student’s *t*-Test
	Mean	SD	Mean	SD	Mean	SD	
r^2^	0.99139	0.00279	0.99252	0.00248	0.98801	0.00461	ns
y0	−76.24995	2.09408	−76.72142	1.18568	−74.37373	3.29214	ns
A1	32.20208	21.07782	75.13608	70.93642	21.86118	2.22605	ns
t1	428.35330	382.32851	230.65180	188.23041	395.76677	44.87687	ns
A2	20.39047	0.80461	31.85999	9.43239	21.95694	2.03324	ns
t2	488.72723	289.74814	193.88591	160.66524	395.76430	44.87630	ns
A3	27.83466	13.65964	148.00675	188.50018	21.98332	2.02220	ns
t3	645.22967	156.50354	168.40045	156.08010	395.75803	44.87675	* (for MASMC v/s sEND1)

**Notes:** Statistical significance is indicated as ns (not significant). *p-value < 0.05, **p-value < 0.01 and ***p-value < 0.001.

For LIDE (Table 1), the differences in r^2^ value between MASMC, sEND1 or co-culture were not significant (ns). This indicated that the exponential decay function was an equally good fit for the curves with the different cell types. The curve fitting parameter t_2_ was significantly different (p < 0.01) for MASMC v/s sEND1. This indicated that the parameter t_2_ could be used to distinguish between these 2 cell types. For SIDE (Table 2), the differences in r^2^ value between MASMC, sEND1 or co-culture were not significant (ns). This indicated that the exponential decay function was an equally good fit for the curves with the different cell types. The curve fitting parameter t_3_ was significantly different (p < 0.05) for MASMC v/s sEND1. This indicated that the parameter t_3_ could be used to distinguish between these 2 cell types.

**Figure 10:** Experimental Mean Impedance per unit area vs Mean Phase data and fitted curves for Large IDE with MASMC (**A**), sEND1 (**B**) & co-culture (**C**) and Small IDE with MASMC (**D**), sEND1 (**E**) & co-culture (**F**).

The Mean impedance per unit area vs Mean phase plots in this paper cannot be compared to results from other papers, as this electroanalytical plot has never been previously used. However, using Log Resistance v/s Log Reactance plots, Bagnaninchi and Drummond demonstrated a clear difference in complex impedance trace between osteo-induced and adipo-induced stem cells, following induction. The main limitation of their study is that the complex impedance trace prior to induction was not shown. Using Nyquist diagrams, Teixeira et al demonstrated a clear difference between L929 cells and HaCaT cells. L929 showed only one dispersion while HaCaT showed 2 dispersions, indicated by 2 semi-circles. The limitation of their study is that the error bars were not shown on the diagrams, and it is thus not clear whether this was a reproducible result. My results show that the MIPUA vs Mean phase plots can provide a reproducible and visually obvious method of distinguishing between a pure smooth muscle cell monolayer and a pure endothelial monolayer, and between a pure endothelial cell monolayer and a co-culture. Moreover, AUC analysis provided a statistical method of characterising the different monolayers. The main limitation is that this method was not tested with other different cell types. Further experiments are required with other cell types to determine whether they generate curves which are significantly (visually and statistically) different from that of MASMCs and sEND1. If different cell types do generate significantly different MIPUA vs Mean Phase curves, then a library of “signature spectra” for could be generated for “electrical characterisation” of cells.

The article "Characterising Vascular Cell Monolayers Using Electrochemical Impedance Spectroscopy and a Novel Electroanalytical Plot" was retracted in 2021. Reasons: no approval from the institution; no approval from a third party; a breach of policy by an author.

This novel method of electrical characterisation of vascular cells could be valuable in engineered vascular grafts. It could be used to non-invasively determine whether endothelial cell only and smooth muscle cells only are located in the inner and outer layers of the engineered grafts, prior to implantation. However, the electrical characterisation was only carried out using 2D cell monolayers, and it is not clear whether this method would be applicable to 3D tubular structures. In this paper, the 2-electrode technique was used to measure the electrical impedance spectra, as it is very sensitive to the cell monolayer directly in contact with the electrodes.^32^ Due to the masking effect of the first layer, the electrodes become less sensitive to cells above the monolayer, making the 2-electrode technique inappropriate for multi-layered or 3D structures. The 4-electrode technique is sensitive to cells across several layers and to biomass density. Further works will focus on a combination of 2-electrode and 4-electrode EIS to characterise multi-layered or 3D vascular tissue.

## Conclusions

This paper reports on a novel electroanalytical diagram (mean impedance per unit area vs mean phase) which can be used for the “electrical characterisation” of cell monolayers consisting of smooth muscle cells, endothelial cells or co-culture. Conventional Bode diagrams are not suitable for characterising different cell monolayers, as different cell types generate impedance spectra with identical shapes. MIPUA vs Mean phase plots can provide a reproducible and visually obvious method of characterising cell monolayers. Additionally, the AUC analysis showed that the difference was statistically significant. Their results cannot be compared to results from other papers, as this electroanalytical plot has never been previously used. However, Bagnaninchi and Drummond and Teixeira et al have used similar approaches, and demonstrated that different cell types generated different complex impedance spectra. The results in this paper are reproducible as 3 technical replicates and different electrode dimensions were used. Miniaturising the interdigitated electrodes increases the cell detection capability and monolayer characterisation capability. Fitting a “Three-phase exponential decay function with time constant parameters” onto the MIPUA vs Mean Phase curve was a promising quantitative method of characterising these curves. The curve fitting parameters t_2_ and t_3_ were significantly different for the MASMC v/s sEND1 data acquired using LIDE and SIDE, respectively.

The article "Characterising Vascular Cell Monolayers Using Electrochemical Impedance Spectroscopy and a Novel Electroanalytical Plot" was retracted in 2021. Reasons: no approval from the institution; no approval from a third party; a breach of policy by an author.

Further work is required to determine whether this method could be extended to other cell types, and if this is the case, a library of “signature spectra” could be generated for “electrical characterisation” of cells. This could complement other well-established cell characterisation methods. Further work is also required to determine whether this novel electroanalytic plot could be generated using both the 2-electrode and 4-electrode impedance measurement technique. This would then enable characterisation of multi-layered and 3D.
